This article has been retracted.

# The Determination of Efficacy of CircuCare on Blood Circulation and Metabolism: An Animal Model Study

**DOI:** 10.1155/2021/9934107

**Published:** 2021-12-02

**Authors:** Kai-Ting Chien, Ching-Chen Chen, Chien-Ming Chu, Ya-Lin Chan, Hsiu-Yun Chung, Ting-Kuo Chang

**Affiliations:** ^1^Department of Orthopaedic Surgery, Mackay Memorial Hospital, Taipei, Taiwan; ^2^L.D.Y. Clinic of Chinese Medicine, New Taipei City, Taiwan; ^3^Biomedical Development Center, Mackay Memorial Hospital, Taipei, Taiwan; ^4^Animal Centre, Mackay Memorial Hospital, Taipei, Taiwan; ^5^Department of Orthopedic Surgery, Mackay Memorial Hospital, Taipei, Taiwan

## Abstract

**Objectives:**

To determine whether feeding CircuCare to rats improves blood circulation, metabolism, immune regulation, endocrine activity, and oxidative stress.

**Methods:**

28 eight-week-old male Sprague-Dawley rats were evenly randomized into control and experimental groups. The control group was fed with ordinary drinking water, while the experimental group was fed with CircuCare at a daily dose of 93.75 mg per 300 g of body weight over eight weeks. Both groups were subjected to a swimming test, and blood samples were taken to observe any variations in various biochemical parameters before and after the test. *Key Findings*. The experimental group's mean swimming exhaustion duration was 53.2% longer and had a significantly higher lactic acid removal ratio. Their mean prostaglandin E2 level and mean glucose, cortisol, and glutathione level (30 minutes after swimming test) were also significantly higher. No undesirable impacts from CircuCare relating to general blood biochemistry values and bone mineral density were reported.

**Conclusions:**

The present results show that CircuCare can be safely used to increase stamina and exercise capability, expedite the metabolism of lactic acid, accelerate muscle repair, and promote the antioxidant activity of cells in rats.

## 1. Introduction

The proper blood flow in the circulatory system is critical to the maintenance of life, as it supplies nutrients to cells throughout the body, in addition to enabling gas exchange, the transport of metabolites, and the maintenance of homeostasis [1]. The causes of insufficient blood circulation include aging, diseases (such as diabetes), unhealthy lifestyle (such as smoking and poor diets), and accidental injuries [2–6]. According to existing literature, a variety of symptoms may result from insufficient blood circulation, such as cold extremities, mental exhaustion, and sore and numb limbs. Poor blood circulation can even induce stroke and cardiovascular disease in severe cases [7–11].

CircuCare (DC Botanical Biotechnology Co., Ltd.) is a traditional Chinese medicine (TCM) that has some unique properties. It is a herbal product that is intended to boost metabolism; improve blood circulation and so-called “*qi*” deficiency; eliminate soreness, numbness, swelling, and pain; and enhance blood circulation to dissipate blood stasis. The major ingredients of this herb product consist of papaya, *Acanthopanax senticosus* (Rupr. et Maxim.) Harms, Chinese fevervine, Chinese Angelica, Panax ginseng C.A. Meyer, red dates, and licorice. These ingredients are chosen on the basis of the TCM theory regarding the compatibility of “monarch, minister, assistant, and guide” herbs [12].

According to the Chinese Pharmacopeia and related TCM literature, papaya and Panax ginseng C.A. Meyer are “monarch” medicines and thus the main active ingredients of CircuCare, with papaya helping in relaxing the muscles, protecting the vascular network, and removing dampness to restore normal functioning of the stomach. Panax ginseng C.A. Meyer replenishes vital energy and cardiac function [13–15]. The Chinese fevervine and *Acanthopanax senticosus* (Rupr. et Maxim.) Harms, present in CircuCare, act as “minister” medicines helping in fortifying the effects of monarch medicines. Chinese fevervine is intended to help the papaya expediting the removal of metabolic waste from the muscles and blood vessels. *Acanthopanax senticosus* (Rupr. et Maxim.) Harms is intended to aid the Panax ginseng C.A. Meyer in boosting the immunity and stamina of the body. The Chinese Angelica acts as an “assistant” medicine to boost the efficacy of the formulated prescription, with the specific aim of enriching the blood and promoting blood circulation, thus helping to improve vascular perfusion and inhibit platelet activity to reduce the risk of thrombosis. The red dates and licorice act as “guide” medicines, which exercise a harmonizing effect among the various other types of medicine [13–15].

With these intended effects in mind, the present study is conducted on rats feeding with Chinese herb compound to determine its efficacy in improving blood circulation, metabolism, immune regulation, endocrine activity, and oxidative stress.

## 2. Materials and Methods

### 2.1. Experimental Animals and Groups

A total of 28 eight-week-old male Sprague-Dawley (SD) rats purchased from BioLASCO Taiwan Co., Ltd. were used in the experiments, with 14 rats each randomized into the control group and the experimental group. Each rat weighed around 300 g at the start of the experiments. The rats were weighed every week. The standard feeds provided to the experimental group and the control group were equal in terms of calories, proteins, and fat. Otherwise, the rats in the control group were fed with ordinary drinking water, while those in the experimental group were fed with CircuCare at a dose of 93.75 mg per 300 g of body weight per day, with the sample feeding period lasting for eight weeks (that is, 40 days, with no feeding on Saturdays and Sundays). The dose provided was calculated on the basis of the bioavailability of a rat being 6.25 times more than that of a human [16]. The absorption rate and metabolic rate of CircuCare in the rats, however, were not investigated in this study.

The rats in both groups were subjected to a swimming test to evaluate the difference of exercise endurance between two groups. Blood samples were also taken from the rats in order to observe any variations in the values of various biochemical parameters before and after the swimming test exercise and, in turn, to determine whether CircuCare expedited the elimination of metabolic waste from the bodies of the experimental group rats after the exercise. The mice were transported to and euthanized in their home chambers; i.e., euthanasia chambers were constructed of clear material and free of debris and excreta. During the euthanization process, CO_2_ was gradually introduced into the chambers at a flow rate of 10-20% of the chamber volume per minute. Once all the mice became unconscious, the flow rate was increased to hasten the process. In summary, the experiments were conducted to understand and analyze the improvement in blood circulation, metabolism, immune regulation, endocrine activity, and oxidative stress based on the experimental results for the swimming test and blood samples. The experimental process of the study is shown in Figure 1, and the content and purpose of each test performed are described below.

### 2.2. Swimming Training and Endurance Test

The rats in both groups were subjected to a swimming endurance test based on the protocol previously described by Chu [17]. Briefly, after having been fed for four weeks, the rats in both groups were required to engage in brief bouts of swimming training for the next four weeks (that is, from week 5 through week 8). Specifically, the rats were subjected to a 15-minute swimming session thirty minutes after being fed three times per week. Then, at 30 to 60 minutes after being fed at the end of week 8, each rat was placed in a glass water tank with a diameter of 20 cm, a depth of 50 cm, and a water temperature maintained at 25 ± 1°C. Each rat was forced to swim and struggle until its energy was completely consumed and it sank. This was the swimming endurance test. For each rat, the time from being placed in the water to the end of seven consecutive seconds during which the head of the rat remained beneath the surface of the water was recorded. In order to evaluate the stamina of the rats, each rat had iron weights placed on its back during the experiment so that it constituted a weight-bearing swimming test. The total weight used for each rat was around 10% of the rat's body weight.

### 2.3. Serum Biochemistry Tests and Blood Lactic Acid Ratio Tests

Blood was collected from the tail vein of each rat for a blood biochemistry analysis of blood urea nitrogen (BUN), glucose, cortisol, glutathione (GSH), and prostaglandin E_2_ (PGE2) levels at four different periods of time, namely, before the experiment, after four weeks of feeding, before the swimming endurance test, and then after the rat was sacrificed following the swimming endurance test. Blood was also collected to determine the blood lactic acid ratio of each rat at three different periods of time, namely, shortly before the swimming test, 10 minutes after the swimming test, and 30 minutes after the swimming test.

For the blood lactic acid ratio test, after the blood was treated, the enzyme action and colorimetric assay principles were applied with lactate oxidase added into a fixed amount of plasma for reaction, followed by the addition of 4-aminoantipyrine and 1,7-dihydroxynaphthalen. Under the action of peroxidase, red compounds were generated. The absorbance was determined at a wavelength of 540 nm before the concentration of lactic acid was obtained. The lactic acid values obtained before and after the swimming test were used to calculate the ratio of elevation in lactic acid. Meanwhile, the lactic acid removal ratio was calculated using the values at 10 minutes and 30 minutes after the swimming. With the lactic acid elevation/removal ratio, one can infer the effect of CircuCare on the generation of lactic acid during exercise (as a result of fatigue) and its effect on the rate at which postexercise lactic acid is metabolized (resulting in the elimination of fatigue).

Taken together, that biochemical parameters tested in the serum blood biochemistry and lactic acid ratio tests provide a range of physiological information. Specifically, blood glucose and lactic acid are both indicators of acute biochemical metabolism, which can cause the consumption of sugar and the formation of lactic acid to occur during exercise. BUN, a metabolite of protein, is eliminated from the body in urine after being secreted by the kidneys, such that elevated BUN levels indicate abnormal kidney function. Cortisol, a hormone secreted by the adrenal gland, is an indicator of endocrine stress (or “stress hormone”) that increases blood pressure and blood sugar levels and gives rise to immunosuppressive effects, with a normal level of cortisol helps in maintaining the body's internal balance in response to stress. PGE2 is an inflammatory factor, and studies have indicated that when an inflammatory response or muscle damage occurs, the synthesis of PGE2 is increased and may, therefore, play an important role in muscle repair [18]. GSH is an important antioxidant in the human body and was used herein as an antioxidant blood biochemistry indicator.

### 2.4. Micro-Computed Tomography (CT) Imaging

In order to determine whether CircuCare is helpful for bone growth, a micro-CT imaging device (Bruker SKYSCAN 1176, Belgium) was used after the swimming endurance test and final blood draw to measure several parameters of each rat's femur, including the bone mineral density (BMD), bone volume (BV), trabecular number (Tb.N), trabecular separation (Tb.Sp), and trabecular bone thickness (Tb.Th), with the resulting measurements subjected to analysis.

### 2.5. Statistical Analysis

The BMD, BV, Tb. N, Tb.Sp, Tb.Th, and swimming time of the rats in the control and experimental groups were compared using the independent sample *t*-test. For the other dependent variables with repeated measures, including the body weight and glucose, BUN, cortisol, PGE2, GSH, and lactic acid levels, the effect of the intervention was assessed using a generalized estimating equation (GEE) model. Each GEE model included the main effects of the intercept, group (1 = experiment; 0 = control), and measurement (time points as a categorical variable), and the two-way interactions of group × measurement. A significant two-way interaction indicated a significant difference in the change from baseline to a later time point between the control and experimental groups. In addition, the difference for each dependent variable between the control and experimental groups at each time point was also assessed using the simple main effect within the GEE model. All tests were 2-tailed, and *P* < 0.05 was considered statistically significant. No adjustment of multiple testing (multiplicity) was made in this study. Data analyses were conducted using SPSS 25 (IBM SPSS Inc., Chicago, Illinois).

## 3. Results

The cross-sectional-dependent variable results of the rats in the experimental and control groups are shown in Figure 2. No significant differences in BMD, BV, Tb.N, Tb.Sp, or Tb.Th were observed between the two groups (Figures 2(a)–2(e)). However, the rats in the experimental group had a significantly longer mean swimming time than did the control rats (213 sec. vs. 139 sec., *P* = 0.007; Figure 2(f)) for the swimming endurance test conducted after 8 weeks from the start of the intervention.

Figure 3 shows the body weight distribution for each study group across the weekly measurements. The results indicated that the mean body weight of the control group rats increased by a significantly greater amount from the baseline measurement to the first week follow-up measurement than did the mean body weight of the experimental group rats (*B* = −9.72, *P* = 0.001; Figure 3). However, the increases in weight from the baseline to the 2nd through 8th weeks were similar for the experimental group and control group.

The changes in mean glucose level from the baseline to week 4 and from the baseline to week 8 before the swimming endurance test were similar for the two groups. However, a significantly greater increase in the glucose level from the baseline to week 8 after the swimming endurance test was observed in the control group (*B* = −27.7, *P* < 0.001; Figure 4(a)). In addition, the mean glucose level of the control group at week 8 after the swimming was significantly higher than that of the experimental group (*P* < 0.05). With respect to BUN levels, the rats in the experimental group exhibited a significantly lower increase from the baseline to week 8 before the swimming endurance test than did the rats in the control group (*B* = −2.03, *P* = 0.018; Figure 4(b)). Meanwhile, there were no significant cortisol level differences between the two groups in terms of either the changes between measurements or the mean at each measurement (Figure 4(c)).

With respect to PGE2 levels, there was a greater increase from the baseline to week 8 week after the swimming endurance test in the experimental group (*B* = 1.98 × 10^3^, *P* = 0.006; Figure 4(d)). In addition, the PGE2 level of the experimental group at week 8 after the swimming test was significantly higher than that of the control group (*P* < 0.05). With regard to GSH levels, the experimental group demonstrated a significantly greater increase from the baseline to week 8 after the swimming test than did the control group (*B* = 2.27, *P* = 0.004; Figure 4(e)). Furthermore, the GSH level of the experimental group at week 8 after the swimming test was significantly higher than that of the control group (*P* < 0.05). With respect to lactic acid levels, the increase from shortly before the swimming test to 10 minutes after the swimming was greater in the experimental group than in the control group (*B* = 4.30, *P* = 0.016; Figure 4(f)). Moreover, the lactic acid level at 10 minutes after the swimming was also significantly higher in the experimental group than in the control group (*P* < 0.05).

## 4. Discussion

In TCM, *qi*, which has been translated variously as “life force,” “energy flow,” “material energy,” and similar phrases, is regarded as the vital force of any living organism [19, 20]. Relatedly, TCM theory holds that various illnesses and symptoms are due to imbalances, deficiencies, or disruptions of *qi* in the organs or meridians and that these imbalances can be alleviated by correcting the flow of *qi* through various means, including the administration of herbal medications [21]. The related concepts of *yin* and *yang* refer not only to the duality of opposing but also complementary and interconnected forces, with TCM theory holding that a balance between the *yin* and *yang* qualities within the body is required for good health [22, 23]. TCM theory further holds that various herbs are able to balance *qi*, *yin*, and *yang* by dint of their specific effects, and past studies have supported a variety of positive effects from different ingredients used in TCM formulations, including those used in CircuCare.

With respect to the monarch medicines included in CircuCare, a number of studies have indicated that Panax ginseng C.A. Meyer can have positive physiological effects. For example, a recent study by Kim et al. found that Panax ginseng C.A. Meyer had antifatigue effects in humans who engaged in anaerobic exercise, while an earlier study of dexamethasone-treated rats by Lin et al. found that Panax ginseng C.A. Meyer significantly decreased their alanine aminotransferase (ALT) and aspartate aminotransferase (AST) levels, suggesting liver protective effects, in addition to restoring the adrenal and thyroid functions inhibited by dexamethasone [24–26]. Meanwhile, previous studies have indicated that papaya has positive cardiovascular and hypertension-related effects in rats [27, 28].

Past studies have also found positive effects from Chinese fevervine and *Acanthopanax*, the minister medicines included in CircuCare, with a study by Yan et al. finding Chinese fevervine to have potent hypouricemic activity in rats and a study by Kato et al. finding that the increased concentrations of lactate in the blood after high-intensity exercise were reduced by *Acanthopanax senticosus* (Rupr. et Maxim.) Harms, suggesting that the herb has an antifatigue effect [29, 30]. Meanwhile, Chinese Angelica, mixed in CircuCare as an additive, was found to be resulted in reduced serum lactate, ammonia, and creatine kinase levels in mice that are subjected to exercise, resulting in enhanced exercise performance and reduced fatigue compared to control mice not treated with the herb [24]. Finally, the guide medicines included in CircuCare, red dates and licorice, have been found to enhance the expression of antioxidant enzymes and neurotrophic factors in cultured astrocytes (suggestive potential benefits to the brain) and to provide a wide range of medicinal effects, including antitussive, anti-inflammatory, and antibacterial effects, among others [31, 32].

The findings of those previous studies support the results of the present study. First, the results indicated that CircuCare provided a number of functional improvements for the rats treated with it. Specifically, the experimental group rats showed a mean swimming exhaustion duration 53.2% longer than that of the control rats (*P* < 0.01), while the lactic acid removal ratio of the experimental rats was also significantly higher than that of the control rats (*P* < 0.05), meaning that the lactic acid metabolism rate of the experimental rats was quite high, approximately twice than that of the control rats. This implied that experiment rats had better exercise endurance and fast recovery than control rats, which may contribute by the effect of Panax, *Acanthopanax senticosus* (Rupr. et Maxim.) Harms, and Chinese Angelica. Furthermore, the mean PGE2 level of the experimental rats was obviously increased compared to that of the control group rats (*P* < 0.05), indicating that the synthesis of PGE2 was significantly increased, potentially expediting muscle repairs. Lastly, the mean GSH level of the experimental rats at 30 minutes after the swimming test was significantly higher than that of the control group (*P* < 0.05), suggesting that the experimental group rats were conserving the use of GSH, which has been inferred to promote the antioxidant activity of cells. Such effect may result from the ingredients of red dates and licorice.

Meanwhile, with respect to safety, the mean body weights of the experimental group and control group rats increased consistently over each week of the experiment, with no statistically significant differences between the two groups. There were likewise no other indications of undesirable impacts from CircuCare in the experimental group rats in terms of changes in their general blood biochemistry values (liver and kidney functions) or BMD as compared to those in the control group. Taken together, these weight, biochemistry, and BMD results suggest that CircuCare can be used safely.

## 5. Conclusion

In summary, the results of the present study indicate that CircuCare can be safely used to increase stamina and exercise capability, expedite the metabolism of lactic acid, accelerate muscle repair, and promote the antioxidant activity of cells in rats without causing any undesirable impacts. These results suggest that CircuCare can be safely applied to humans for the similar benefits. Further research can validate this possibility.

## Figures and Tables

**Figure 1:** Experimental flowchart of the study: (1) plasma biomarker test, (2) lactic acid ration test, (3) swimming exhaustion test, and (4) micro-CT scan.

**Figure 2:** Comparisons between the control group and experimental group in terms of bone volume (a), trabecular thickness (b), trabecular separation (c), trabecular number (d), bone mineral density (e), and swimming time (f). In each graph, the horizontal lines indicate the means, and the error bars indicate the standard errors of the means.

**Figure 3:** Body weight measurements of the control group and experimental group at the baseline and weekly follow-ups. At each time point, the horizontal lines indicate the means, and the error bars indicate the standard errors of the means. The “‡” symbol indicates a significant difference between the two groups in the change from the baseline to the indicated time point.

**Figure 4:** Comparisons between the control group and experimental group across time points in terms of glucose (a), BUN (b), cortisol (c), PGE2 (d), GSH (e), and lactic acid (f) levels. In each graph, the horizontal lines indicate the means, and the error bars indicate the standard errors of the means. The “‡” symbol indicates a significant difference between the two groups in the change from the baseline to the indicated time point. The “∗” symbol indicates a significant difference between the two groups for the means measured at a specific time point.

## Data Availability

The datasets used and/or analyzed during the current study are available from the corresponding author on reasonable request.

## Abbreviations

ALT: Alanine aminotransferase
AST: Aspartate aminotransferase
BMD: Bone mineral density
BUN: Blood urea nitrogen
BV: Bone volume
GEE: Generalized estimating equation
GSH: Glucose, cortisol, glutathione
PGE2: Prostaglandin E2
SD: Sprague-Dawley
Tb.N: Trabecular number
Tb.Sp: Trabecular separation
Tb.Th: Trabecular bone thickness
TCM: Traditional Chinese medicine.
